The article "Identification of MicroRNA Targeting Mlph and Affecting Melanosome Transport" was published in 2019. Journal: Biomolecules.

# Identification of MicroRNA Targeting *Mlph* and Affecting Melanosome Transport

**DOI:** 10.3390/biom9070265

**Published:** 2019-07-08

**Authors:** Jeong Ah Lee, Seok Joon Hwang, Sung Chan Hong, Cheol Hwan Myung, Ji Eun Lee, Jong Il Park, Jae Sung Hwang

**Affiliations:** Department of Genetic Engineering & Graduate School of Biotechnology, Kyung Hee University, Yongin, Gyeonggi-do 446-701, Korea

**Keywords:** melanosome transport, melanophilin, microRNA

## Abstract

Melanosomes undergo a complex maturation process and migrate into keratinocytes. Melanophilin (Mlph), a protein complex involving myosin Va (MyoVa) and Rab27a, enables the movement of melanosomes in melanocytes. In this study, we found six miRNAs targeting *Mlph* in mouse using two programs (http://targetscan.org and DianaTools). When melan-a melanocytes were treated with six synthesized microRNAs, miR-342-5p, miR-1839-5p, and miR-3082-5p inhibited melanosome transport and induced melanosome aggregation around the nucleus. The other microRNAs, miR-5110, miR-3090-3p, and miR-186-5p, did not inhibit melanosome transport. Further, miR-342-5p, miR-1839-5p, and miR-3082-5p decreased *Mlph* expression. The effect of miR-342-5p was the strongest among the six synthesized miRNAs. It inhibited melanosome transport in melan-a melanocytes and reduced *Mlph* expression in mRNA and protein levels in a dose-dependent manner; however, it did not affect Rab27a and MyoVa expressions, which are associated with melanosome transport. To examine miR-342-5p specificity, we performed luciferase assays in a mouse melanocyte-transfected reporter vector including *Mlph* at the 3′-UTR (untranslated region). When treated with miR-342-5p, luciferase activity that had been reduced by approximately 50% was restored after inhibitor treatment. Therefore, we identified a novel miRNA affecting *Mlph* and melanosome transport, and these results can be used for understanding Mlph expression and skin pigmentation regulation.

## 1. Introduction

Melanocytes, a type of skin cell, produce melanin and are located in the basal layer of the epidermis. Melanin is a biological pigment comprising the reddish-yellow type called pheomelanin and the brownish-black type eumelanin [1,2]. The differences in skin color among individuals from different races result from the type of melanin produced and not from the number of melanocytes [3].

Melanosomes are lysosome-related organelles that produce, store, and transport melanin, and result in the pigmentation in melanocytes [4]. The transport of mature melanosomes from the perinuclear area to the dendrite tips of melanocytes is facilitated by microtubule- and actin-dependent motor proteins [5]. Actin-dependent melanosome transport is associated with the tripartite complex proteins, Rab27a, melanophilin (Mlph), and myosin Va (MyoVa). Rab27a is a GTPase and a member of the Ras oncogene family, and its effector molecule is Slac2-a/Mlph, which recruits the actin-dependent motor protein MyoVa [5,6,7]. Defects in melanosome transport cause a condition known as Griscelli syndrome (GS). Griscelli and colleagues found two girls with skin hypopigmentation and silver-gray hair [8]. There are three types of GS, GS types 1, 2, and 3, caused by mutations in MyoVa, Rab27a, and Mlph, respectively [9]. All three types cause skin and hair hypopigmentation; however, GS types 1 and 2 cause neurological impairment and immunological impairment, respectively, as side effects. However, with Mlph mutation, only depigmentation is reportedly apparent and no other side effects are observed [10,11,12]. Therefore, *Mlph* could be an important target gene for depigmentation studies.

The roles of many uncharacterized miRNAs in the skin have been studied. For example, miR-31 enhances cell proliferation and migration in keratinocytes, and aids in skin wound healing [13]. A previous study showed that miR-218 decreased melanogenesis by directly inhibiting microphthalmia-associated transcription factor (MITF) in melan-a mouse melanocytes [14]. Recent studies targeted the 3´-UTR of genes associated with melanosome transport. For example, miR-203 significantly suppressed the growth of human and canine melanoma cells and inhibited melanosome transport through the suppression of MITF and Rab27a expressions [15]. In addition, miR-145 reportedly decreases MyoVa and FSCN1 expressions in human melanoma cells [16]. However, miRNAs that only target *Mlph* among the motor proteins associated with melanosome transport in mouse melanocytes have not yet been reported. In this study, we attempted to find miRNAs that regulate *Mlph* expression.

## 2. Results

### 2.1. Identification of miRNAs Targeting Mlph in Mice

To identify miRNA targeting *Mlph* in mice, we used two programs. One was TargetScan, and the other was DIANA-microT v3.0. These two online bioinformatics programs predicted miRNAs that could directly target the 3′-UTR of *Mlph*. In all, 265 miRNAs were predicted by TargetScan and 17 by DIANA-microT v3.0. We synthesized six miRNAs and inhibitors (Inh) identified by both programs (Figure 1). The microRNA sequences are shown in Table 1.

### 2.2. Effect of miRNAs on Mlph Expression in Melan-a Melanocytes

To investigate whether the six synthesized miRNAs affect melanosome transport, melan-a mouse melanocytes were treated with 10 nM of the miRNAs. After 72 h transfection, we found that melanosome aggregation was induced. Three miRNAs, miR-342-5p, miR-3082-5p, and miR-1839-5p, induced melanosome aggregation in melan-a melanocytes. However, the other three did not induce melanosome aggregation (Figure 2a). Among the six miRNAs, miR-342-5p had the strongest inhibitory effect on the Mlph protein expression level compared to the negative control (Figure 2b).

### 2.3. Effect of miR-342-5p on Mlph Expression in Melan-a Melanocytes

To investigate whether miR-342-5p affected melanosome transport in a dose-dependent manner, miR-342-5p was treated with 2.5 nM, 5 nM, and 10 nM miR-342-5p for 72 h (Figure 3a). Treatment with 2.5 nM, 5 nM, and 10 nM miR-342-5p increased melanosome aggregation in a dose-dependent manner compared with control. miR-342-5p decreased the mRNA and protein levels of *Mlph* in a dose-dependent manner (Figure 3b,c). The mRNA *Mlph* expression level was measured using quantitative real-time PCR.

The aggregation of melanosomes around the nucleus was imaged using HMB45 antibody immunofluorescence (Figure 3d).

### 2.4. Effect of mir-342-5p on the Rab27a and MyoVa Expressions

To determine whether miR-342-5p affects other key melanosome transport protein expressions, we examined Rab27a and MyoVa expressions together. miR-342-5p decreased the level of Mlph but did not affect the levels of MyoVa and Rab27a. To check the specificity of the effect of miR-342-5p on Mlph expression, the rescue effect was examined using an inhibitor of miR-342-5p (Figure 4a). The inhibitor of miR-342-5p increased the levels of Mlph.

### 2.5. miR-342-5p Directly Targets Mlph in Melan-a Melanocytes

We identified the binding site of mmu-miR-342-5p in the 3´-UTR of *Mlph* (Figure 4b). To identify the specificity of miR-342-5p, we constructed a sensor vector by joining the 3′-UTR region of mouse *Mlph* to a luciferase reporter pGLuc-basic vector. To determine the target sequence recognized by the miRNA, miR-342-5p was treated with an inhibitor, while the control was not. Treatment with miR-342-5p reduced luciferase activity, and treatment of miR-342-5p with inhibitor restored the luciferase activity (Figure 4c).

## 3. Discussion

Melanosomes are fully matured during transport from the melanocyte nucleus to the melanocyte dendrite tip. Then, melanosomes are transferred to the keratinocytes [17,18]. During melanosome transport, three proteins, Mlph, Rab27a, and MyoVa, form a tripartite complex. These are the key regulators of melanosome transport [19,20].

In this study we identified miRNAs that affected Mlph expression, and attempted to understand their effect. When the melan-a melanocytes were treated with the selected miRNAs, the miRNAs were observed to suppress melanosome transport (Figure 2a). Significant aggregation of melanosomes in the perinuclear area was evident in the transfection of miR-342-5p in melan-a melanocytes (Figure 3a). miR-342-5p decreased the protein levels of Mlph in a dose-dependent manner (Figure 3b). Previous studies have showed that miR-5110 suppresses pigmentation in alpaca melanocytes by co-targeting MLPH and WNT family member 1 [21]. However, miR-5110 has no effect on melanosome transport in melan-a melanocytes. miR-342-5p decreased the levels of Mlph, but did not affect Rab27a and MyoVa expressions (Figure 4a). Until now there has been no report on the miRNA targeting *Mlph* in mice or humans. From this study, we found miRNA that affects the expression of Mlph in mice, and we can expect miRNAs with similar function in humans, which is an area of research to be explored in future studies. According to several previous studies, Mlph expression is very important for melanosome transport. Mutations in *Mlph* have been shown to cause defects in melanosome transport in melanocytes [7]. Treatment with miR-342-5p reduced the mRNA level of Mlph (Figure 3c) by targeting the 3´-UTR of Mlph.

miR-3082-5p and miR-1839-5p downregulated Mlph and Rab27a expression levels (data not shown). There are reports that one miRNA can target two genes simultaneously. For example, a study published in Japan in 2013 showed that one miRNA can target two genes simultaneously in a gastric cancer cell line [22]. miR-224 targets DPYSL2 (dihydropyri-midinase-like-2) and KLAS, which is a proto-oncogene [22]. DPYSL2 encodes the collapsin response mediator protein 2 (CRMP2), a cytosolic protein [23]. This protein is necessary for the growth and promotion of neurons. It is usually tethered to the cell membrane, and is essential for tissue signaling. Therefore, miR-3082-5p and miR-1839-5p can be considered to target two genes simultaneously, similar to miR-224. miR-3082-5p is reportedly controlled in mouse melanoma cells by curcumin and could be a potential anti-cancer miRNA [24]. However, miR-1839-5p has not yet been investigated.

It has been reported that miR-342-5p is upregulated in Alzheimer’s disease (AD) transgenic mouse models, including APP/PS1, PS1DE9, and PS1-M146V lines [25]. miR-342-5p binds directly to the 3’-UTR of AnkG mRNA and decreases AnkG levels through translation repression in AD transgenic mouse neurons. However, there have been no reports on the effects of miR 342-5p on Mlph expression. We found a novel miRNA that affects Mlph and melanosome transport and could be important for understanding Mlph expression and skin pigmentation regulation.

## 4. Materials and Methods

### 4.1. Materials

miRNA was purchased from GenePharma (Shanghai, China). Lipofectamine RNAi MAX was purchased from Invitrogen (Carlsbad, CA, USA).

### 4.2. Cell Culture

Melan-a melanocytes are highly pigmented, immortalized murine melanocytes derived from C57BL/6 mice. Melan-a melanocytes were obtained from Dr. Dorothy Bennett (St. George’s Hospital, London, UK). Melan-a melanocytes were maintained in RPMI-1640 medium (Welgene, Gyeongsan, Korea) supplemented with 10% fetal bovine serum (FBS), 10 U/mL penicillin, 100 μg/mL streptomycin, and 200 nM phorbol 12-myristate 13-acetate (PMA; Sigma-Aldrich Co., St. Louis, MO, USA).

### 4.3. Transfection

One day before transfection, melan-a melanocytes were seeded in six-well plates at 60% confluency, and miRNAs, inhibitors, and 20 nM siRNA mixed RNAi MAX (Invitrogen) were applied according to the manufacturer’s protocol.

### 4.4. Western Blotting

Blots were incubated with β-actin antibody (1:20000, Sigma), MyoVa antibody (1:800, Cell Signaling Technology, Beverly, MA, USA), Rab27a antibody (1:500, Santa Cruz, CA, USA), Mlph antibody (1:800, ProteinTech Group, Inc. Chicago, IL, USA) at 4 °C overnight. Blots were then washed three times with TBS-T (Tris Buffered Saline with Tween 20) and incubated with horseradish peroxidase-conjugated anti-rabbit (1:1000, Bethyl Laboratories, Montgomery, AK, USA) or anti-mouse (1:20000, Bio-Rad, Hercules, CA, USA) antiserum at room temperature for one hour. Bound antibodies were detected using a SuperSignal® West Pico Chemiluminescent Substrate (Thermo Scientific, Waltham, MA, USA). The bands on the membranes were detected via chemiluminescence and visualized with FluorChem E (ProteinSimple, San José, CA, USA).

### 4.5. Immuno-Fluorescence (IF)

One day before transfection, melan-a melanocytes were seeded in one chamber at 60% confluency and miRNA plus 20 nM siRNA mixed RNAi MAX (Invitrogen) were applied according to the manufacturer’s protocol. Melan-a melanocytes transfected with miRNA and siRNA after 72 h were washed with DPBS (Dulbecco’s Phosphate-Buffered Salin) and then were fixed in 2 mL formalin for 15 minutes at room temperature. Chambers were washed three times with PBS and were then permeabilized with 1 mL of 0.1% Tripton for 15 minutes and then blocked using 1 mL of 2% BSA(Bovine Serum Albumin). After thorough washing, sections were incubated with first antibody (HMB45) diluted with 2% BSA for two to three days at 4 °C with shaking. FITC-conjugated antibody was diluted 2% BSA or PBS treated for one hour at 4 °C with shaking followed by washing three times with PBS. The cells were stained with 4′-6-diamidino-2-phenylindole DAPI) for 15 minutes at room temperature.

### 4.6. Quantitative Real-Time PCR

Quantitative real-time PCR was performed using a FastStart Essential DNA Probe Master kit (Roche, Mannheim, Germany) with the Universal Probe Library (Roche). The reaction was carried out according to the manufacturer’s protocol. The probes for Rab27a (#21, NM_023635.5), *Mlph* (#108, NM_053015.3), and MyoVa (#21, NM_010864.2) were designed using the Probe Library Assay Design Center. The cycling conditions were 600 seconds at 95 °C followed by 40 cycles at 95 °C for 20 seconds and 60 °C for 40 seconds on a Lightcycler® Nano (Roche, Basel, Switzerland). The resulting cDNA was amplified with the following primers: Rab27a sense 5′-GAAGACCAGAGGGCAGTGAA-3′, and antisense 5′-ACTGGTTTCAAAA-TAGGGGATTC-3′; MyoVa sense 5′-GCGCCATCACCCTAAACA-3′, and antisense 5′-CCAGTTGACTGACATTGTACCTG-3′. The three gene expression levels were normalized to mouse β -actin.

Values are presented as mean ± SD from three wells.

### 4.7. miRNA and Small Interfering RNAs

To investigate potential miRNAs targeting melanophilin, we used two programs, TargetScanMouse (http://www.targetscan.org) and Diana Tools (http://diana.imis.athenainnovation.gr/DianaTools/index.php).

All miRNA used in this study, including inhibitors for each microRNA, were purchased from GenePharma (Shanghai, China) (Table 1). siRNA oligonucleotides were purchased from Bioneer (Daejeon, Korea). Sense and antisense sequences for individual duplexes targeting mouse *Mlph* were as follows: *Mlph* sense was 5’-GGGCAAAAUACAAAAGGAGUUTT–3’, and antisense was 5’- CUCCUUUUGUAUUUUGCCCUUTT–3’.

### 4.8. Detection and Quantification of Melanosome Aggregation

Melan-a melanocytes were seeded in 24-well plates and cultured for 24 h. The cells were then rinsed in DPBS and treated with samples of RPMI- 1640 containing 2% FBS for three days. The cells were observed under bright field using a digital microscope (iRiS^TM^, Logosbio, Korea). Evaluation of melanosome aggregation was performed by counting cells with perinuclear melanosome aggregates in three random microscopic fields per well at 200× magnification.

Values are presented as mean ± SD from three wells.

### 4.9. Luciferase Assay

We constructed a sensor vector by joining the regions with a possible binding site from the 3′-UTR of mouse *Mlph* to a luciferase reporter pGLuc-basic vector purchased from Cosmogenetech (Seoul, Korea) in order to identify the target sequences recognized by the miRNAs. For amplification of these mRNAs, melan-a melanocytes were seeded in six-well plates at a concentration of 3.0 × 10^5^/well the day before the transfection. The vector, at a concentration of 0.5 μg/well, and 10 nM miRNAs or nonspecific control miRNA was used for the co-transfection of the cells using the cationic liposomes Lipofectamine RNAi MAX. Luciferase activities were measured using a BioLux Luciferase Assay Kit (NEW ENGLAND BioLabs Inc., MA, USA) according to the manufacturer’s protocol, 48 h after the cotransfection.

## Figures and Tables

**Figure 1:** Prediction of miRNAs targeting melanophilin (*Mlph*) in mice.

**Figure 2:** Effect of miRNAs in melan-a melanocytes. Melan-a melanocytes were seeded at 3 × 10^5^ cells/well in 10π dishes in RPMI-1640 media with 10% FBS(Fetal Bovine Serum), 1% P/S, and 200 nM TPA. (**A**) After 24 h, melan-a melanocytes were treated with miRNAs. We examined cells transfected with six representative microRNAs. After 72 h, the cells were observed in bright field using a digital microscope (iRiS^TM^, Logosbio, Anyang, Korea). Melanosome aggregation was estimated by counting cells with perinuclear melanosome aggregation in three random microscopic fields per well at 200× magnification. (**B**) Melan-a melanocytes treated with 10 nM miRNAs for 72 h. Six miRNAs showed effects on protein expression level from Mlph. Values are presented as the mean ± SD from three wells.

**Figure 3:** Effects of miR-342-5p in melan-a melanocytes. Melan-a melanocytes were seed at 3 × 10^5^ cells/well in 10π dishes in RPMI-1640 media with 10% FBS, 1% P/S, 200 nM TPA. (**A**) After 24 h, melan-a melanocytes were treated with miR-342-5p in a dose-dependent manner. After transfection for 72 h, the cells were observed in bright field using a digital microscope (iRiS^TM^, Logosbio, Korea). (**B**) Melan-a melanocytes treated with 10 nM miRNAs for 72 h. miR-342-5p effects on the level of Mlph. (**C**) Cells were harvested for RNA 48 h after transfection. *Mlph* expression levels were determined using real-time q-PCR. The experiment was repeated three times. Data were analyzed using Student’s un-paired *t*-test **, *p* < 0.01. (**D**) Melan-a melanocytes were seeded at 2 × 10^5^ cells/chamber. After 24 h, melan-a melanocytes were treated with miRNA and siRNA according to the manufacturer’s protocol. After 72 h, cells were photographed. Values are presented as the mean ± SD from three wells.

**Figure 4:** Mlph, MyoVa, and Rab27a expression levels by miR-342-5p or with inhibitors. Melan-a melanocytes were seeded at 3 × 10^5^ cells in six-well plates for 24 h. (**A**) After 24 h, melan-a melanocytes were treated with miR-342-5p and inhibitors. After 72 h, miR-342-5p effected the levels of Mlph, MyoVa, and Rab27a. (**B**) We examined whether mmu-miR-342-5p directly targets *Mlph* by using online miRNA target prediction databases. (**C**) Luciferase reporters were linked with *Mlph* 3‘-UTRs. miR-342-5p or scrambled mimic (Scr mimic) were co-transfected with a luciferase-UTR construct into melan-a melanocytes, and luciferase activity was determined.

**Table 1:** Sequences of microRNAs used in this study.

microRNA	Sequence
miR-1839-5p	5’-AAGGUAGAUAGAACAGGUCUUG-3’
miR-5110	5’-GGAGGAGGUAGAGGGUGGUGGAAUU-3’
miR-3082-5p	5’-GACAGAGUGUGUGUGUCUGUGU-3’
miR-342-5p	5’-AGGGGUGCUAUCUGUGAUUGAG-3’
miR-3090-3p	5’-UCCCAGGUGACACCCUGACUCA-3’
miR-186-5p	5’-CAAAGAAUUCUCCUUUUGGGCU-3’
miR-1839-5p Inh.	5’-CAAGACCUGUUCUAUCUACCUU-3’
miR-5110 Inh.	5’-AAUUCCACCACCCUCUACCUCCUCC-3’
miR-3082-5p Inh.	5’-ACACAGACACACACACUCUGUC-3’
miR-342-5p Inh.	5’-CUCAAUCACAGAUAGCACCCCU-3’
miR-3090-3p Inh.	5’-UGAGUCAGGGUGUCACCUGGGA-3’
miR-186-5p Inh.	5’-AGCCCAAAAGGAGAAUUCUUUG-3’
